# Construction of Biologic Microscopic Image Segmentation Model Based on Smoothing of Fourth-Order Partial Differential Equation

This article has been retracted.

**DOI:** 10.1155/2022/1908644

**Published:** 2022-07-25

**Authors:** Ye Ma

**Affiliations:** Department of Biomedical Engineering, Jilin Medical University, Jilin, China 132013

## Abstract

In order to solve the problem of microscopic image noise, a biological microscopic image segmentation model based on the smoothing of the fourth-order partial differential equation was proposed. Based on the functional description of image smoothness by directional curvature mode value, a fourth-order PDE image denoising model is derived, which can effectively reduce noise while preserving edges. The result of this method is piecewise linear image, and the gradient at the edge of the target has a step. Using the feature of noise reduction, a new geodesic active contour model is proposed. The experiment result shows that when the variance of Gaussian white noise is 15, the enhancement and denoising effects of the proposed method are 80.35% and 69.84 higher than those of the original vibration filtering method and L. Alvarez method. In terms of time, the proposed method is 1.3075 seconds slower than the original vibration filtering method and 17.5754 seconds faster than the L. Alvarez method. When the variance of Gaussian white noise is 25, the enhancement and denoising effects of the proposed method are 97.79% and 81.16 higher than those of the original vibration filtering method and L. Alvarez method. In terms of time, the proposed method is 1.3246 seconds slower than the original vibration filtering method and 17.5796 seconds faster than the L. Alvarez method. *Conclusion*. The new model is not only stable but also has strong ability of contour extraction and fast convergence.

## 1. Introduction

Medical imaging is an important part of the noninvasive diagnostic process implemented by today's healthcare systems. It involves the creation of visual and functional representations of the body's interior and organs for clinical analysis. Medical imaging technology is mainly divided into imaging based on X-ray (examples include traditional x-rays, computed tomography (CT), and mammography), microimaging, magnetic resonance imaging (MRI), ultrasound (US), and optical coherence tomography (OCT). Based on these medical imaging technologies, various types of biomedical images are increasingly being used to diagnose various diseases [1]. Medical imaging consists of two parts: (1) image formation and reconstruction and (2) image processing and analysis. Image formation involves the process of forming a two-dimensional (2D) image of a three-dimensional (3D) object, while image reconstruction relies on a set of iterative algorithms, usually forming two-dimensional and three-dimensional images from projected data of the object. Image processing, on the other hand, involves the use of algorithms to enhance the properties of the image, such as noise removal, while image analysis extracts quantitative information or a set of features from the image for target identification or classification, such as medical image segmentation techniques [2].

In the field of computer vision, image segmentation refers to the process of dividing an image into multiple regions. The goal of segmentation is to simplify and/or change the representation of the image, making it more meaningful and easier to analyze [3]. Some of the practical applications of image segmentation include medical imaging to study anatomical diagnosis, treatment planning or locating tumors, and other pathological diagnoses. In addition, image segmentation technology is also widely used in face recognition, machine vision, satellite target positioning, and other fields, as shown in Figure 1.

## 2. Literature Review

Özdür et al. combined the excellent time-frequency localization characteristics of wavelet in the field of filtering and denoising with the threshold method to overcome the influence of noise in cell images. This method has a good segmentation effect on simple adhesions of quasicircular cells (adhesions of less than 3 cells), but poor segmentation effect on complex adhesions of irregular shape cells [4]. Chen et al. proposed a multithreshold segmentation method for cell images; that is, cell images are segmented into multiple regions by using gray distribution. This method is effective when there is a significant difference between two adjacent regions of the target in the image, but when the cell edge is blurred and the gray distribution of the image is seriously uneven, the segmentation result is not satisfactory [5]. Inspired by the features, Li et al. proposed a multithreshold segmentation algorithm of color histogram with block overlapping for cell graphs stained under the microscope, although this method is better than the traditional color histogram segmentation method. However, it is necessary to update a histogram with a large color change in real time and calculate the Euclidean distance between the reference model and the reference model, which requires a large amount of calculation and is difficult to ensure the segmentation efficiency and robustness to the light [6]. Liu et al. used Delaunay triangulation to divide the cell image into irregular triangles [7]. Chen et al. noted that in addition to dividing the cell image horizontally and vertically, the image was also split in two at 45 and 275 directions [8]. In order to solve the problem of fixed segmentation location, Wang and Chen chose the optimal location to achieve horizontal or vertical segmentation. The above algorithms do not take into account the actual boundary shape of cells but artificially divide the image into some fixed shapes and approach the boundary of cells by constantly subdividing the shapes, which is easy to produce block effect or oversegmentation at the edge of cells [9]. Nlü and Kiri proposed a cell segmentation method based on Sobel operator for the feature of strong speckle noise in the image of gastric adenocarcinoma cells. This method suppressed the speckle noise by making cursive changes to the image, but the edge continuity detected by Sobel operator was not good, and the edge was easy to miss detection when the gray difference between cells and background was small [10]. Liu et al. proposed a method of calculating the segmentation of oval cells. On the basis of ROI extraction and Canny operator's preliminary detection of cell edges, Gauss conic curve fitting was used to accurately locate cell edges. This method has a good segmentation effect on elliptic cells, but not on irregular shape cells [11].

Image noise has a great influence on the segmentation effect of active contour model, especially for the edge based model. Therefore, the regional global partition method is introduced into the region-based model to partially solve this problem. But in some cases, image smoothing pretreatment is still needed. In this paper, the directional curvature mode is used to measure the image smoothness, and a method of biological microscopic image smoothness based on the fourth-order partial differential equation is derived from the functional. The result of this method is a piecewise linear image, and there is a step in the gradient of the target edge. Experimental results show that the proposed denoising method can greatly improve the segmentation effect of both edge- and region-based active contour models.

## 3. Research Method

### 3.1. Design and Image Acquisition of Fluorescence Microscopic Imaging System Based on Structured Light Illumination

#### 3.1.1. Principle of Fluorescence Microscopic Imaging

High-performance fluorescence microscopic imaging system (including automatic focusing platform) provides high-quality cell images for subsequent postprocessing of medical microscopic cell images, which is the premise and key of medical microscopic cell image segmentation in this paper. This section is the key and core content of the whole article [12].

As a kind of optical microscope, fluorescence microscope plays an important role in biomedical research. Fluorescence microscopy uses fluorescence molecules as probes to label biological tissues and obtain spatial information of samples by detecting the distribution of fluorescence signals emitted by excited fluorescence molecules. When a substance is irradiated by a light wave with a shorter wavelength, it emits a light with a longer wavelength, as shown in Figure 2. The energy of phosphorescence is lower than that of fluorescence, so its wavelength is longer than that of fluorescence, and its life span can reach several hours. Excitation materials emit fluorescent light called excitation light; its spectrum includes ultraviolet blue light and has been extended to yellow-green light band [13].

The process of fluorescence is the interaction between light and matter. Fluorescent groups (fluorescent substances probe dye proteins, etc.) that stain cell samples absorb excitation light at a specific central wavelength and undergo an energy-level transition from the ground state to the excited state. Then, the Stokes shift occurs, the frequency shifts to the intermediate state, and finally, the transition back to the lower energy order (ground state) and the emission of fluorescent photons (emission of light). Due to the Stokes frequency shift, the energy of the emitted fluorescent photon is lower than that of the excited photon; that is, the wavelength of the emitted light is longer than that of the excited light.

#### 3.1.2. How Fluorescence Microscopy Works

Fluorescence microscope based on fluorescence characteristics has the basic structure of optical microscope and optical magnification; it also has the following unique properties: high fluorescence contrast, selective excitation, high sensitivity, and the red shift of the signal light relative to the excitation light (which is conducive to the separation of the signal light and the excitation light). These unique features improve the image quality of the optical microscope [14]. Given the Stokes shift, how do you build a fluorescence microscope that irradiates a sample at a single wavelength, filters out the light reflected back, and only sees the fluorescence with a longer wavelength shift?

In fact, it is very similar to how George Gabriel Stokes first noticed fluorescence: a purple glass window allegedly filtered sunlight onto a bottle of tonic water, which he then observed was filled with white wine, blocking out the purple light. The preferred method of modern fluorescence microscopy is surface illumination, that is, falling fluorescence microscopy, which uses an objective lens to illuminate and image the sample. An upright microscope with a slide at the bottom, in this case the light source, is an arc lamp that sends full-spectrum light to the sample through a fluorescent cube that selectively illuminates the sample with the wavelength that excites the particular fluorophore [15]. The excited red fluorescence sends photons in all directions, some of which are collected by the objective and sent to the camera port above through the cube which has two filters, a dichromatic mirror and a barrier filter, to prevent the excited wavelength from reaching the detector.

In this structure, the microscope objective not only has the usual role of imaging and magnifying the sample but also acts as a condenser to illuminate the sample. The advantage of this approach over transmission fluorescence microscopy (in which the excited light passes through the condenser and the emission is collected by the objective) is that, although the excitation of the fluorophore is the same as that of the transmission microscope, only a small portion of the excited light reflected from the sample needs to be blocked in the return path in the fall-illumination mode.

The main technical obstacle of falling fluorescence microscopy is the overlapping of excitation light and fluorescence emission in the light path, which requires a special beam splitter, namely, dichromatic mirror, to separate excitation and emission. The design of dichromatic beam splitter uses a 45-degree light path. In an ordinary fluorescence microscope, dichromatic mirror reflects the light from the source at shorter wavelengths and transmits the longer wavelengths of the fluorescence emitted. Each dichromatic mirror is designed to have a transition from reflection to transmission between the excitation and emission peaks of the fluorophore for which it is designed. Dichromatic mirrors are rarely used without two additional filters: an excitation filter with a preselected excitation wavelength and a barrier filter that only allows light of longer wavelengths to return to the detector. All three of these filters are typical interference filters with very specific wavelength selectivity, and these are engineering marvels made up of many thin stacks of materials with alternating refractive indices. With the exciter beam splitting bicolor circuit and the barrier circuit, these three components can be very good separation of excitation light and emitted light.

### 3.2. Image Smoothing Based on Fourth-Order Partial Differential Equation

The image function *I* is regarded as the surface defined in the three-dimensional space (*x*, *y*, *I*(*x*, *y*)), as shown in Figure 3. Specify a point *p* and a direction $\overset{⟶}{d}$ on *I*, and then, the change of the normal vector of the surface of the point *p* in the direction $\overset{⟶}{d}$ is expressed by the directional curvature $\overset{⟶}{n}$. Directional curvature is a second-order description of the change speed of the surface along the tangent direction of a certain point on the surface, which can quantitatively express the change of the surface around a certain point:

(1) $$\begin{array}{c} m^{2}=0.5\cdot \left(I_{xx}^{2}+I_{yy}^{2}\right)+I_{xy}^{2}. \end{array}$$

Thus, we consider the following defined functional over the region as shown in

(2) $$\begin{array}{c} E\left(I\right)=\int_{\Omega }\;F\left(m^{2}\right)\text{d}x\text{d}y. \end{array}$$

*m* ^2^ is shown in equation (1) and *I* ∈ *C*^4^(*Ω*). Function *F*(·) ≥ 0 is an increasing function, namely, *F*′(·) > 0. The operator *m*^2^ can describe the roughness of the local surface. Therefore, the larger the roughness (noise) of the image surface *I* is, the larger the functional value of equation (2) is, and the minimization of *E*(*I*) is equivalent to image smoothness [16]. Euler equation about equation (2) is obtained by using variational method:

(3) $$\begin{array}{c} \left.\frac{\partial^{2}}{\partial x^{2}}\left(F^{\prime }\left(m^{2}\right)I_{xx}\right)+2\frac{\partial }{\partial x\partial y}\left(F^{\prime }\left(m^{2}\right)I_{xy}\right)+\frac{\partial }{\partial y^{2}}F^{\prime }\left(m^{2}\right)I_{y}\right)=0. \end{array}$$

Euler equation shown in formula (3) can be solved by gradient descent method as shown in

(4) $$\begin{array}{c} \frac{\partial I}{\partial t}=\&-\left[\frac{\partial^{2}}{\partial x^{2}}\left(F^{\prime }\left(m^{2}\right)I_{xx}\right)+2\frac{\partial^{2}}{\partial x\partial y}\left(F^{\prime }\left(m^{2}\right)I_{xy}\right)+\left.\frac{\partial^{2}}{\partial y^{2}}\left(F^{\prime }\left(m^{2}\right)I_{yy}\right)\right]\right.. \end{array}$$

The conduction function is shown in

(5) $$\begin{array}{c} F^{\prime }\left(m^{2}\right)=\frac{1}{1+m^{2}/K^{2}}. \end{array}$$

 *K* is threshold of conductivity coefficient; selecting different *K* values can control the retention and smoothing of different image features. The original image is taken as the input, and the final solution *t*⟶∞ is obtained at that time so that the image is not overly smooth; the iteration must be terminated within a limited time.

The image whose gray function satisfies the plane equation is a linear image. Obviously, when the image *I* is a linear image, the gradient $\nabla I=\left(\partial_{I}/\partial_{x}\right)\overset{⟶}{i}+\left(\partial I/\partial_{y}\right)\overset{⟶}{j}$ is constant. Laplace ∇^2^*I* evaluates to zero and the operator *m*^2^ = 0.5 · (*I*_*xx*_^2^ + *I*_*yy*_^2^) + *I*_*xy*_^2^ is zero, so that the left end of equation (3) is equal to

(6) $$\begin{array}{c} F^{\prime }\left(0\right)\left(I_{xxxx}+2I_{xxyy}+I_{yyy}\right)=F^{\prime }\left(0\right)\left(\frac{\partial^{2}}{\partial x^{2}}\left(I_{xx}+I_{yy}\right)+\frac{\partial^{2}}{\partial y^{2}}\left(I_{xx}+I_{yy}\right)\right)=F^{\prime }\left(0\right)\left(\frac{\partial^{2}}{\partial x^{2}}\left(\nabla^{2}I\right)+\frac{\partial^{2}}{\partial y^{2}}\left(\nabla^{2}I\right)=0\right.. \end{array}$$

It can be seen that the linear image satisfies Euler equation (3), and since the function *F*(·) is nonnegative, the functional *E*(*I*) satisfies

(7) $$\begin{array}{c} E\left(I\right)\geq 0. \end{array}$$

At the same time, the function *F*(*m*^2^) is an increasing function, and the global minimum is obtained when the linear image *m*^2^ = 0 is drawn, that is, the global minimum of the functional.

Other minima may exist in the functional *E*(*I*), and we show that piecewise linear images satisfy Euler's equations.

Set *Ω*_*i*_, *i* = 1, 2, ⋯, *n* as the division of image region, and the piecewise linear image is shown in

(8) $$\begin{array}{c} I\left(x,y\right)=\overset{n}{\underset{i=1}{\sum }}\;I_{i}\left(x,y\right), \end{array}$$

where,

(9) $$\begin{array}{c} I_{i}\left(x,y\right)=\left\{\begin{array}{c} \text{ planar image},\left(x,y\right)\in \Omega_{i},\\ 0. \end{array}\right. \end{array}$$

*I*_*i*_ ∈ *C*^4^(*Ω*_*i*_); the composite image *I*(*x*, *y*) should be continuous. Any two adjacent images *I*_*i*_, *I*_*j*_ shown in formula (9) must satisfy different plane equations; otherwise, they can be combined. *∂Ω*_*i*_ is the boundary of area *Ω*_*i*_; *Ω*_*i*_ − *∂Ω*_*i*_ is the internal part of *Ω*_*i*_, satisfying the following equations:

(10) $$\begin{array}{c} \nabla I_{i}\left(x,y\right)=\text{constant }\left(x,y\right)\in \left(\Omega_{i}-\partial \Omega_{i}\right), \end{array}$$

(11) $$\begin{array}{c} \nabla^{2}I_{i}\left(x,y\right)=0, \end{array}$$

Therefore, the algorithm is shown in

(12) $$\begin{array}{c} \begin{array}{c} \nabla^{2}I\left(x,y\right)=0,\\ m^{2}\left(x,y\right)=0.5^{\circ }\left(I_{xx}^{2}+I_{yy}^{2}\right)+I_{xy}^{2}=0. \end{array} \end{array}$$

(*x*, *y*) ∈ (*Ω* − *∂Ω*), *∂Ω* = ⋃_*i*=1_^*n*^ *∂Ω*_*i*_. Since any two adjacent *I*_*i*_ and *I*_*j*_ sums are on different planes, the gradient at the boundary *∂Ω* is discontinuous, as shown in

(13) $$\begin{array}{c} \nabla I_{i}\neq \nabla_{I_{j}}. \end{array}$$

As shown in formula (14),

(14) $$\begin{array}{c} \nabla^{2}I\left(x,y\right)=\infty ,\left(x,y\right)\in \partial \Omega . \end{array}$$

For the operator *m*^2^(*x*, *y*), the calculation formula is shown in

(15) $$\begin{array}{c} m^{2}=\frac{1}{2}\left(I_{xx}^{2}+I_{yy}^{2}\right)+I_{xy}^{2}=\frac{I_{xx}^{2}+I_{xy}^{2}+I_{yy}^{2}+I_{xy}^{2}}{2}\geq \frac{2I_{xx}I_{xy}+2I_{yy}I_{xy}}{2}=I_{xy}\left(I_{xx}+I_{yy}\right)=I_{xy}\nabla^{2}I. \end{array}$$

(*x*, *y*) ∈ *∂Ω*. If *I*_*xy*_ equals to zero, then the calculation method is shown in

(16) $$\begin{array}{c} \begin{array}{c} m^{2}=\frac{1}{2}\left(I_{xx}^{2}+I_{yy}^{2}\right)+I_{xy}^{2}=\frac{I_{xx}^{2}+I_{yy}^{2}}{2},\\ {\left(\nabla^{2}I\left(x,y\right)\right)}^{2}=\infty =I_{xx}^{2}+I_{yy}^{2}+2I_{xx}I_{yy}\leq 2\left(I_{xx}^{2}+I_{yy}^{2}\right). \end{array} \end{array}$$

So we get

(17) $$\begin{array}{c} m^{2}=\frac{1}{2}\left(I_{xx}^{2}+I_{yy}^{2}\right)+I_{xy}^{2}=\infty . \end{array}$$

The result is shown in

(18) $$\begin{array}{c} F^{\prime }\left(\infty \right)=0. \end{array}$$

If *I*_*xx*_ equal to infinity (∞), then the calculation method is shown in

(19) $$\begin{array}{c} F^{\prime }\left(m^{2}\right)I_{xx}=\frac{1}{\left(1/I_{xx}\right)+\left(\left(\left.0.5*\left(I_{xx}+I_{yy}^{2}/I_{xx}\right)\right)+I_{xy}^{2}/I_{xx}\right)/K^{2}\right)}=0. \end{array}$$

It is a similar case for *I*_*xx*_ and *I*_*yy*_.

Therefore, when it is a piecewise linear image, the result is shown in

(20) $$\begin{array}{c} \begin{array}{c} \left.\frac{\partial^{2}}{\partial x^{2}}\left(F^{\prime }\left(m^{2}\right)I_{xx}\right)+2\frac{\partial^{2}}{\partial x\partial_{y}}\left(F^{\prime }\left(m^{2}\right)I_{xy}\right)+\frac{\partial^{2}}{\partial y^{2}}F^{\prime }\left(m^{2}\right)I_{yy}\right)=0,\\ \left(x,y\right)\in \Omega . \end{array} \end{array}$$

It can be seen that the segmented linear image satisfying Euler equation (formula (4)) is the noise reduction model of the fourth-order partial differential equation derived in this paper [17].

### 3.3. New Geodesic Active Contour Model Based on Smoothing of Fourth-Order Partial Differential Equation

Geodesic active contour (GAC) proposed by Caselles et al. is a model based on curve evolution theory and level set method. It can deal with topological structure changes of curve movement freely without any external control conditions, and it is the most widely used edge model [18].

Geodesic active contour identifies image features (such as edges) with functions *g*(*I*) and was aimed at minimizing energy functions. The motion equation of the corresponding contour curve *C* is shown in

(21) $$\begin{array}{c} \frac{\partial C}{\partial t}=g\left(I\right)\left(k+V_{0}\right)\overset{⟶}{N}-\left(\nabla g\left(I\right)\cdot \overset{⟶}{N}\right)\overset{⟶}{N}, \end{array}$$

where *k* is the curvature of the curve, $\overset{⟶}{N}$ is the normal unit vector of the curve, *V*_0_ is the constant, and *g*(*I*) takes a minimum value at the edge, as shown in

(22) $$\begin{array}{c} g\left(I\right)=\frac{1}{1+{\left|\nabla \left[G_{\sigma }*I\right]\right|}^{2}}, \end{array}$$

where *G*_*σ*_ represents the two-dimensional Gaussian filter operator with the standard deviation of *σ* and ∗ is the convolution operator.

The last term *g*(*I*) is edge attraction, which is an image force pointing towards the edge of the image. When the curve moves near the target edge, this term applies an external force pointing towards the edge of the curve, thus pulling the curve towards the target. In the actual image processing, the target edge is not the ideal edge, and it is not zero at the edge *g*(*I*). At this point, the curve motion stops near the target by the balance of the edge attraction and the force of the first term, so the target positioning performance is limited [19].

On the basis of image smoothing by the denoising model derived in this paper, we propose a new edge identification function as shown in

(23) $$\begin{array}{c} G\left(I\right)=\frac{1}{1+{\left|\nabla^{2}I\right|}^{2}}. \end{array}$$

The corresponding new geodesic active contour (NEW-GAC) model is shown in

(24) $$\begin{array}{c} \frac{\partial C}{\partial t}=g\left(I\right)\left(k+V_{0}\right)\overset{⟶}{N}-\left(\nabla G\left(I\right)\cdot \overset{⟶}{N}\right)\overset{⟶}{N}. \end{array}$$

As we know from the above, different images *K* can be selected to control the smoothness of image features, and the smoothed image is a piecewise linear image with a step in the gradient at the target edge, as shown in

(25) $$\begin{array}{c} \nabla^{2}I\left(x,y\right)=\infty ,\left(x,y\right)\in \partial \Omega . \end{array}$$

Therefore, the new edge identification function can better achieve the effect of the ideal geodesic active contour model. In the experimental results, we will see that compared with the traditional geodesic active contour model, the new geodesic active contour model proposed in this paper is more ideal in edge positioning.

## 4. Interpretation of Result

In order to verify the effect of the proposed method in image enhancement and denoising, the synthetic images and brain images with different variances of Gaussian white noise and salt and pepper noise were selected for enhancement and denoising. The original vibration model, L. Alvarez method model, and the method in this paper are used to process the noise image, and the results are compared [20, 21].

The results of image enhancement and denoising of Gaussian white noise and appropriate amount of salt and pepper noise are given when the number of iterations is 100. It is obvious that the vibration filtering equation can enhance the image and amplify the noise signal at the same time. The L. Alvarez method has some effect on image enhancement and denoising. However, when the noise is large, the original image structure cannot be well maintained, and the sharp corner information is seriously lost. Compared with the previous two methods, the method in this paper has a better effect, and the original image structure is relatively intact, and the sharp corner information is also well maintained [22, 23].

The enhancement and denoising results of several methods in medical images are given, in which the variance of the image noise is 15 Gaussian white noise, and the number of iterations is 15. It can be seen from the figure that the processing effect of the method in this paper is significantly better than that of the first two methods, which not only enhances the image and removes the noise but also maintains more image details.

In this paper, peak signal-to-noise ratio (PSNR) is also used as the enhancement and denoising effect measurement index. PSNR reflects the statistical average of image signal-to-noise ratio changes. It is a widely used method to measure the subjective quality of images. The greater the PSNR, the better the image quality and the worse the image quality. As shown in Figures 4–7, it can be seen that the effect obtained by using this algorithm is superior to other methods when the variance of Gaussian white noise is 15. The enhancement and denoising effects of the proposed method are 80.35% and 69.84% higher than those of the original vibration filtering method and L. Alvarez method. In terms of time, the proposed method is 1.3075 seconds slower than the original vibration filtering method and 17.5754 seconds faster than the L. Alvarez method. When the variance of Gaussian white noise is 25, the enhancement and denoising effect of the proposed method is 97.79% and 81.16% higher than that of the original vibration filtering method and L. Alvarez method. In terms of time, the proposed method is 1.3246 seconds slower than that of the original vibration filtering method and 17.5796 seconds faster than that of L. Alvarez method. At the same time, we give the calculation time of various algorithms in the composite image and find that the time of the method in this paper is much smaller than that of the method, mainly because the linear smooth Gaussian kernel *G*_*σ*_ is no longer used to denoise the vibration item in each iteration [24, 25].

## 5. Conclusion

This paper proposes a functional to describe the image smoothness based on the directional curvature mode value and then deduces a fourth-order PDE image denoising model. The processing result is piecewise linear image (including linear image), and the gradient at the edge has a step. In this paper, a new geodesic active contour (NEW-GAC) model is proposed, which improves the contour extraction performance of the original vibration filtering method and the L. Alvarez method with good speed. It is worth noting that NEW-GAC makes full use of the characteristics of the denoising model derived in this paper, and the two methods together constitute a new image segmentation method. The region-based active contour model has some robustness to noise, but the processing of strong noise graph is still limited. The noise reduction model in this paper also greatly improves the segmentation effect of region-based active contour model.

## Figures and Tables

**Figure 1:** A fourth-order partial differential equation-smoothed biomicroscopic image segmentation model.

**Figure 2:** Phosphorescence and fluorescence generation diagram.

**Figure 3:** Schematic diagram of directional curvature.

**Figure 4:** Comparison of synthetic image enhancement and denoising effect measures (Gaussian white noise variance = 15).

**Figure 5:** Comparison of composite image enhancement and denoising effect measures (Gaussian white noise variance = 25).

**Figure 6:** Comparison of image enhancement and denoising effect measures (variance of Gaussian white noise = 15).

**Figure 7:** Comparison of image enhancement and denoising effect measures (Gaussian white noise variance = 25).

## Data Availability

The data used to support the findings of this study are available from the corresponding author upon request.

## References

[1] Ebihara M., Katayama K. (2020). Anomalous charge carrier decay spotted by clustering of a time-resolved microscopic phase image sequence. *The Journal of Physical Chemistry C*.

[2] Du Y., Xiao G., Liu L., Gui Y., Wei D., Yang X. (2020). Study of solidification and microstructure characteristics for aircraft icing. *International Journal of Thermophysics*.

[3] Kim Y. J., Chai Y. (2020). Splitting of concrete with steel, glass fiber-reinforced polymer, and basalt fiber-reinforced polymer bars exposed to mgso_4. *ACI Structural Journal*.

[4] Özdür N. A., Üçel I. B., Yang J., Aydıner C. C. (2020). Residual intensity as a morphological identifier of twinning fields in microscopic image correlation. *Experimental Mechanics*.

[5] Chen Y. M., Chou F. I., Ho W. H., Tsai J. T. (2021). Classifying microscopic images as acute lymphoblastic leukemia by resnet ensemble model and taguchi method. *BMC Bioinformatics*.

[6] Li M., Gao S., Han H., Zhang C. (2021). L 0 optimization using laplacian operator for image smoothing. *Jisuanji Fuzhu Sheji Yu Tuxingxue Xuebao/Journal of Computer-Aided Design and Computer Graphics*.

[7] Liu Y., Ma X., Li X., Zhang C. (2020). Two-stage image smoothing based on edge-patch histogram equalisation and patch decomposition. *IET Image Processing*.

[8] Chen W., Bai J., Gu X., Li Y., Gui Z. (2020). Separation-based model for low-dose CT image denoising. *The Journal of Engineering*.

[9] Wang W., Chen Y. (2022). An accelerated smoothing gradient method for nonconvex nonsmooth minimization in image processing. *Journal of Scientific Computing*.

[10] Nlü R., Kiri R. (2022). Detection of damaged buildings after an earthquake with convolutional neural networks in conjunction with image segmentation. *The Visual Computer*.

[11] Liu L., Wang L., Xu D. (2021). CT image segmentation method of liver tumor based on artificial intelligence enabled medical imaging. *Mathematical Problems in Engineering*.

[12] Zhang Y., Tian Y. (2021). A new image segmentation method based on fractional-varying-order differential. *Journal of Beijing Institute of Technology*.

[13] Renugambal A., Bhuvaneswari K. S. (2021). Kapur's entropy based hybridised WCMFO algorithm for brain MR image segmentation. *IETE Journal of Research*.

[14] Xue J., Wang Y., Qu A., Zhang J., Sun H. (2021). Image segmentation method for Lingwu long jujubes based on improved fcn-8s. *Nongye Gongcheng Xuebao/Transactions of the Chinese Society of Agricultural Engineering*.

[15] Tian Y., Cao X., Li X., Zhang H., Boulatov R. (2020). A polymer with mechanochemically active hidden length. *Journal of the American Chemical Society*.

[16] Fang L., Wang X., Wang L. (2020). Multi-modal medical image segmentation based on vector-valued active contour models. *Information Sciences*.

[17] Lv H., Zhang F., Wang R. (2020). Fuzzy active contour model using fractional-order diffusion based edge indicator and fuzzy local fitted image. *IEEE Access*.

[18] Yan X., Weng G. (2022). Hybrid active contour model driven by optimized local pre-fitting image energy for fast image segmentation. *Applied Mathematical Modelling*.

[19] Palitta D. (2021). Matrix equation techniques for certain evolutionary partial differential equations. *Journal of Scientific Computing*.

[20] Pourghanbar S., Manafian J., Ranjbar M., Aliyeva A., Gasimov Y. S. (2020). An efficient alternating direction explicit method for solving a nonlinear partial differential equation. *Mathematical Problems in Engineering*.

[21] Sharma A., Kumar R., Talib M., Srivastava S., Iqbal R. (2019). Network modelling and computation of quickest path for service-level agreements using bi-objective optimization. *International Journal of Distributed Sensor Networks*.

[22] Jayakumar J., Nagaraj B., Chacko S., Ajay P. (2021). Conceptual implementation of artificial intelligent based e-mobility controller in smart city environment. *Wireless Communications and Mobile Computing*.

[23] Xin L., Chengyu M., Chongyang Y. (2015). Power station flue gas desulfurization system based on automatic online monitoring platform. *Journal of Digital Information Management*.

[24] Huang R., Zhang S., Zhang W., Yang X. (2021). Progress of zinc oxide-based nanocomposites in the textile industry. *IET Collaborative Intelligent Manufacturing*.

[25] Zhang Q. (2021). Relay vibration protection simulation experimental platform based on signal reconstruction of MATLAB software. *Nonlinear Engineering*.

